The article "Microarray and Bioinformatics Analysis of Differential Gene and lncRNA Expression during Erythropoietin Treatment of Acute Spinal Cord Injury in Rats" was retracted in 2023. Reasons: signs of a paper mill; compromised peer review; unreliable results or conclusions.

# Microarray and Bioinformatics Analysis of Differential Gene and lncRNA Expression during Erythropoietin Treatment of Acute Spinal Cord Injury in Rats

**DOI:** 10.1155/2022/4121910

**Published:** 2022-09-02

**Authors:** Haibo He, Hanwen Huang, Panyong Hu, Zhong Chen

**Affiliations:** ^1^Department of Spinal Surgery, University of South China Affiliated Nanhua Hospital No. 336, Dongfeng South Road, Zhuhui District, Hengyang, Hunan, China; ^2^Department of Spinal Surgery, Zhujiang Hospital of Southern Medical University, 253# Industry Road, 510280 Guangzhou, Guangdong, China; ^3^Department of Spinal Surgery, Affiliated Hospital of Guilin Medical University, No. 15, Lequn Road, Guilin, Guangxi Zhuang Autonomous Region, China

## Abstract

**Purpose:**

We performed a genome-wide analysis of long noncoding RNA (lncRNA) expression to identify novel targets for the further study of recombinant human erythropoietin (rhEPO) treatment of acute spinal cord injury (SCI) in rats.

**Methods:**

Nine rats were randomly divided into 3 groups. No operation was performed in group 1. In groups 2 and 3, a laminectomy was performed at the 10th thoracic vertebra, and a contusion injury was induced by extradural application of an aneurysm clip. Group 1 rats did not receive any treatment, group 2 rats received a single intraperitoneal injection of normal saline, and group 3 rats received rhEPO. Three days after injury, spinal cord tissues were collected for RNA-Seq, microarray, differentially expressed genes (DEGs), Gene Ontology (GO) function enrichment, Kyoto Encyclopedia of Genes and Genomes (KEGG) pathway enrichment, and protein-protein interaction (PPI) analyses.

**Results:**

Compared with group 1, 4,446 genes were found to be differentially expressed in group 2. Furthermore, 99 lncRNAs were found to be changed in the injury group. The data indicate that 2,471 mRNAs were upregulated, and 1,975 mRNAs were downregulated in group 2 as compared with group 1. In addition, 45 of the lncRNAs were upregulated, and the other 44 lncRNAs were downregulated. The top 5 upregulated and top 5 downregulated lncRNAs that were different between group 2 and group 1 are shown. The top 5 downregulated and the top 5 upregulated lncRNAs that were different between group 3 and group 2 are shown.

**Conclusion:**

RhEPO treatment alters the expression profiles of the differentially expressed lncRNAs and genes beneficial to the development of new treatments.

## 1. Introduction

Spinal cord injury (SCI) is a global health problem, and each year, there are 15 to 40 acute SCIs per million persons commonly caused by high falls, community violence, recreational activities, and traffic accidents [1]. SCI can lead to serious damage to the nervous system, including quadriplegia and paraplegia, which seriously affect quality of life [2]. The pathophysiological mechanisms of SCI are complex and involve ischemia-reperfusion leading to endothelial dysfunction and vascular permeability changes, which induce a cascade of inflammation and subsequent neuronal death and loss of neurological function [3].

Although much research has been devoted to elucidate the complex pathophysiological processes that follow SCI, no definitive treatments have been developed. Early decompression surgery can have a positive impact on outcomes. The only pharmacological treatment that is known to ameliorate neurologic dysfunction after SCI is methylprednisolone (MP). Therefore, new therapeutic strategies to promote functional recovery in SCI patients are necessary, and a better understanding of the cellular and molecular mechanisms of SCI may help in the development of new treatments [4].

Erythropoietin (EPO), also known as red blood cell (RBC) stimulating factor, is a human endogenous glycoprotein hormone that stimulates RBC production. The production of EPO is stimulated in a hypoxic environment, and EPO is used clinically for the treatment of anemia associated with renal insufficiency [5]. In a prior study, we reported that recombinant human erythropoietin (rhEPO) reduced apoptosis and inflammation and promoted myelin repair and functional recovery following compressive SCI in rats and that delayed treatment is equally effective [6]. To our knowledge no specific cellular and molecular studies have been undertaken to understand the mechanism by which rhEPO helps repair SCI.

Long noncoding RNAs (lncRNAs) [7] are RNA transcripts longer than 200 nucleotides that lack protein coding ability. Compared to well-studied protein-coding genes, the function of most lncRNAs has not been elucidated, even though a large number of genes have been identified [8, 9]. However, recent studies indicated that lncRNAs are important regulatory molecules in the human genome, which exert their biological control in various ways [10, 11]. lncRNAs have been associated with cell proliferation, survival, and differentiation, genomic stability, and chromatin remodeling [12–14]. With the development of high-throughput sequencing technology, more and more lncRNAs have been identified, and a recent study showed that lncRNA deregulation is an important factor in various nervous system pathologies and that it may play a crucial role in SCI [15].

Thus far, no studies have focused on the differential expression of lncRNAs and mRNAs in SCI treated with EPO. Thus, the purpose of this study was to examine differentially expressed lncRNAs and mRNAs by transcriptome sequencing (RNA-seq) in SCI tissues in a rat model treated with rhEPO. Data from this study may help the development of novel treatments for SCI.

## 2. Materials and Methods

### 2.1. Animals

The study protocols conformed to the Guide for the Care and Use of Laboratory Animals from the National Institutes of Health and were approved by the Animal Care and Use Committee of Southern Medical University. Nine adult male Sprague–Dawley rats (220–260 g) were purchased from the Animal Center of Southern Medical University. All rats were housed 3 per cage under temperature-controlled conditions, with a 12 h light/dark cycle, and had free access to tap water and food.

### 2.2. Experimental Design

The 9 rats were randomly divided into 3 groups: group 1, blank control group; group 2, SCI group; group 3, rhEPO treatment group. All rats were continuously observed and fed for 3 days prior to the experiments.

No procedures were performed on the rats in group 1. They were fed and had free access to water. In group 2, a laminectomy was performed at the 10^th^ thoracic vertebra, and contusion injury was induced by extradural application of an aneurysm clip. The spinal cord was clamped for 30 seconds. Penicillin (1,200,000 U/kg, intramuscular) was given immediately after injury for preventing infection of the surgical incision. An intraperitoneal injection of normal saline (5 ml/kg) was given within 2 hours of the injury and repeated for the next 3 days. Group 3 rats received the same injury as group 2 rats. In group 3, a rhEPO intraperitoneal infusion (3000 U/kg) was given within 2 hours of the injury, and the same rhEPO infusion was given for the next 3 days. As in group 2, penicillin was given immediately after the injury.

Three days after SCI, spinal cord tissue was collected from each rat for the experiments described below.

### 2.3. Surgical Procedures

Rats were deeply anesthetized with an intraperitoneal pentobarbital injection (40 mg/kg) and were fixed in the prone position. Back hair on the surgical area was removed with electric shaver, and the area was disinfected with 3% iodophor. After locating the T10 spinous process, a 2 cm midline incision was made on the midline of the back from the T8 to T12 vertebrae. The overlying musculature was separated laterally, and the spinal cord was exposed by a complete T10 level laminectomy. Subsequently, the spinal cord was subjected to extradural compression with a temporary aneurysm clip (70g force; 65821T; Rebstock, Dürbheim, Germany) for 30 seconds to induce a crush injury. The surgical site was closed using nondegradable sutures after removing the aneurysm clip, and then, the closed skin incision was disinfected again with 3% iodophor. During the procedure, body temperature was maintained with a heat lamp.

After surgery, all rats received 2 ml of 10% glucose solution, tramadol hydrochloride (50 mg/kg) for postoperative analgesia, and penicillin (800,000 U/kg) by intramuscular injection to prevent infection of the surgical incision. The rats were returned to their cages after they completely recovered from anesthesia.

The rats were fed normally with food and water for 3 days, and manual bladder evacuation was performed 3 times a day. On the third postoperative day, the wound was recut and 1 cm of spinal cord tissue was taken from the exposed spinal cord and rapidly frozen in liquid nitrogen. After the sample was completely frozen, it was stored in an airtight container at -80°C until RNA extraction.

### 2.4. RNA Extraction

RNA was extracted from spinal cord tissue using the TRIzol method, according to the manufacturer's instructions.

### 2.5. Microarray Analysis

The mRNA in spinal cord tissue samples was enriched with magnetic beads with the probe named oligo (dT). Subsequently, fragmentation buffer was added to break the mRNA into short fragments, and the mRNA was used as a template to synthesize cDNA using random hexamers. Double-stranded cDNA was then synthesized by the addition of buffer, dNTPs, and DNA polymerase I and RNase H. The double-stranded cDNA was then purified using AMPure XP beads.

Purified double-stranded cDNA was repaired, A-tailed, and ligated to the sequencing linker, and fragment size was selected using AMPure XP beads. Finally, PCR amplification was carried out, and the PCR product was purified with AMPure XP beads to obtain a final library.

After the library was constructed, preliminary quantification was performed using a Qubit 2.0 fluorometer (USA, Invitrogen), and the insert size of the library was subsequently detected using an Agilent 2100 bioanalyzer (USA, Agilent). After the insert was determined to be consistent with expectations, q-PCR was used to accurately quantify the effective concentration of the library to ensure library quality. After the quality of the library was confirmed, the high-throughput sequencing was conducted.

The raw reads, the data by sequencing, need to be filtered to eliminate low-quality reads in order to ensure the quality of the information analysis. The subsequent data obtained is recorded as total data. By removing the known ribosomal RNAs from the total data (28S rRNA, 18S rRNA, 12S rRNA, 5.8S rRNA, and 5S rRNA), high-quality, clean data was obtained. The ribosomal RNA that was removed was identified using the database of the National Center for Biotechnology Information (NCBI, https://www.ncbi.nlm.nih.gov). Subsequent microarray profiling was performed by the Boyue Biotechnology Company (Wuhan, China).

### 2.6. qRT-PCR Validation of Microarrays

To confirm the repeatability of the microarray assays, 6 additional rats were divided into 2 groups and treated the same as the rats in group 2 (SCI group) and group 3 (SCI+rhEPO group), respectively. After total RNA was extracted from the spinal cord of the 6 rats, qRT-PCR assays were performed. Briefly, the qRT-PCR assays consisted of 2 steps, RNA reverse transcription (RT) and qPCR detection. First, the PrimeScript™ RT reagent Kit with gDNA Eraser (TAKARA) was used to synthesize cDNA according to the manufacturer's instructions after removing the genomic DNA. RT-PCR was then performed using SYBR® Premix Ex Taq™ II (TAKARA). The reaction system consists of 10 *μ*l SYBR® Premix Ex Taq™ II, 0.4 *μ*l PCR Forward Primer (10 *μ*M), 0.4 *μ*l PCR Reverse Primer (10 *μ*M), 2 *μ*l cDNA, and 7.2 *μ*l ddH_2_O. The primer sequences were designed and synthesized in the laboratory by the Guangzhou cm biotechnology and are listed in Table 1. The reaction conditions were: 95°C for 10 minutes; a total of 40 cycles at 95°C for 15 seconds and 60°C for 20 seconds. Each sample tested in triplicate. Gene expression levels were normalized to glyceraldehyde 3-phosphate dehydrogenase (GAPDH) using the *ΔΔ*CT method. Finally, Student's *t*-test was used to examine differences between the 2 groups, and values of *p* < 0.05 were considered statistically significant.

### 2.7. Differentially Expressed Gene (DEG) Analysis and Gene Ontology (GO) Enrichment Analysis

DEG analysis refers to the identification of genes with significant differences in expression levels between different sample groups. The clean data was analyzed using the DESeq2 package (http://www.bioconductor.org/packages/release/bioc/html/DESeq2.html) in the R programming language (version 3.60) because our sample had only 3 per group [16]. When the biological repeat reaches 5 to 10, a better choice is to use a nonparametric method.

DESeq2 is the most popular statistical method to analyze DEGs, and it can estimate variance-mean dependence in clean data, and test for differential expression based on a model using a negative binomial distribution. The log2-fold change (log2FC) and *p* values of the genes were calculated [17]. A gene was considered to be a DEG when the log2FC was >1 and the *p* value was <0.05. The lncRNA information was then extracted from DEG analysis result based on the lncRNA annotation information provided in the reference genome annotation file.

GO enrichment analysis is used to annotate genes and gene products and to provide gene function classification labels and background knowledge of gene function and has become a common approach for sequencing data processing [17–19]. GO enrichment analysis can be divided into 3 parts: molecular function (MF), biological process (BP), and cell composition (CC). GO annotation information of genes can be found by searching the GO database by species and genetic information. Based on the GO annotation of a gene, all of the genes of the species can be selected as background genes, and *p* values can be calculated using statistical methods. As such, distribution information and the significance of the gene collection of the GO category can be obtained.

To gain further insights into the changes of biological pathways in the cells of SCI rats, Kyoto Encyclopedia of Genes and Genomes (KEGG analysis) was performed. KEEG is a database of biochemical reactions, signaling pathways, metabolic pathways, and biological processes and can be used to identify the significant pathways associated with DEGs.

The clusterprofiler package (https://bioconductor.org/packages/release/bioc/html/ clusterProfiler.html) in the R programming language (version 3.60) allows 2 methods of analysis. In the analyses in this study, a value of *p* < 0.05 was considered to indicate statistical significance.

### 2.8. Protein-Protein Interaction (PPI) Network Construction

The Search Tool for the Retrieval of Interacting Genes (STRING, http://string-db.org/) is a database that aims to provide a critical assessment and integration of PPI, including direct (physical) and indirect (functional) associations [20]. In the PPI network built using the STRING online tool, each node signifies a gene, and the edges indicate interactions between nodes. The degree is defined as the number of edges linked to a given node.

Cytoscape is software that provides data integration and network visualization [21], especially in respect to the processing of databases of protein-protein interactions [22]. In the current study, the cytoHubba plug-in of Cytoscape (version 3.61) was used to screen the hub genes from the PPI network, and a node degree of ≥10 was screen as the hub genes from the PPI.

## 3. Results

### 3.1. Screening and Identification of DEGs

DEGs between samples were selected by differential multiples (log2FC > 1) and a significance level of *p* < 0.05. Compared with group 1, 4,446 genes were found to be differentially expressed in group 2. Furthermore, 99 lncRNAs were found to be changed in the injury group. The data indicate that 2,471 mRNAs were upregulated, and 1,975 mRNAs were downregulated in group 2 as compared with group 1. In addition, 45 of the lncRNAs were upregulated, and the other 44 lncRNAs were downregulated (Table 2). A volcano plot was created that visually showed how the expressions of the lncRNAs and mRNAs changed dramatically (Figure 1).

A comparison of group 3 with group 2 identified 228 DEGs. Furthermore, 14 lncRNAs were found to be changed in group 3 as compared with group 2 (Table 2).

Cluster analysis of DEGs was used to determine the clustering pattern of DEGs in the different groups. The top 50 genes with the largest variance in expression between the different groups, including the known lncRNAs and mRNAs, were used for cluster analysis (Figure 2).

### 3.2. qRT-PCR

To further confirm the accuracy of the microarray assays, 6 differentially expressed mRNAs, including 3 upregulated mRNAs (Ccl5, Ppbp, and Ahsp) and 3 downregulated mRNAs (Plk5, Mmp7, and Esrp2), were randomly selected for qRT-PCR analysis to compare between group 3 (SCI + rhEPO group) and group 2 (SCI group).

As shown in Figure 3, the expression patterns of the selected mRNAs were consistent with the mRNA-seq results (*p* < 0.05 for each mRNA, Student's *t* test). These results indicated that the microarray were highly reliable.

### 3.3. Top Differentially Expressed lncRNAs between the Groups

The top 5 upregulated and top 5 downregulated lncRNAs that were different between group 2 and group 1 are shown in Table 3. The top 5 downregulated and the top 5 upregulated lncRNAs that were different between group 3 and group 2 are shown in Table 4.

### 3.4. GO and KEGG Pathway Enrichment Analyses

The gene function enrichment analysis was divided into 2 steps: gene function annotation and enrichment analysis. The 3 GO domains used to describe the gene product attributes were MF, BP, and CC (molecular function, biological process, and cell composition, respectively). GO analysis was performed for the DEGs between group 2 and group 1, and the top 15 are shown in Figure 4(a). As shown in the figure, the biological processes of the DEGs were primarily associated with positive regulation of the immune response, regulation of vesicle-mediated transport, regulation of leukocyte activation, wound healing, regulation of transmembrane transport, and other significant biological processes in SCI. In addition, the main 15 KEGG enrichment pathways were related to Epstein-Barr virus infection, focal adhesions, the calcium signaling pathway, retrograde endocannabinoid signaling, osteoclast differentiation, platelet activation, and systemic lupus erythematosus (SLE) and were highly significantly correlated with SCI (Figure 5(a)).

Furthermore, GO and KEGG enrichment analyses were performed between group 3 and group 2 to gain further insights into the changes of biological pathways associated with rhEPO treatment of SCI. GO enrichment analysis reveals 15 significant metabolic networks, including leukocyte chemotaxis, myeloid leukocyte migration, granulocyte migration, granulocyte chemotaxis, neutrophil migration, and other biological processes that were significantly enriched in group 3 (Figure 4(b)). KEGG enrichment analysis indicated that the enriched DEGs were associated with cytokine-cytokine receptor interaction, the chemokine signaling pathway, human cytomegalovirus infection, IL-17 signaling path, malaria, and herpes simplex infection (Figure 5(b)).

### 3.5. PPI Network Construction

Based on data from the STRING database with medium confidence (data chosen had a minimum required interaction score of >0.4), a PPI network with 809 nodes and 5,081 edges was constructed between group 2 and group 1 and was visualized using Cytoscape (Figure 6).

In the PPI network, 10 nodes were selected as hub genes using the Maximal Clique Centrality (MCC) method, which is available in the cytoHubba plug-in of Cytoscape. The hub genes were fibronectin 1 (FN1), protein tyrosine phosphatase receptor type C (PTPRC), cluster of differentiation 4 (CD44), cell division cycle 20 (CDC20), TYRO protein tyrosine kinase-binding protein (TYROBP), aurora kinase B (AURKB), toll-like receptor 2 (TlR2), angiotensinogen (AGT), Rac family small GTPase 2 (RAC2), and matrix metallopeptidase 9 (MMP9). Of the 10 hub genes, FN1 had the highest score of 108 (Table 5).

Similarly, a comparative study of group 3 and group 2 was conducted using the same methods. The constructed PPI network had 70 nodes and 129 edges (Figure 7). The top 10 key genes are shown in Table 6.

## 4. Discussion

In most cases, SCI is a disabling and irreversible disease that is associated with great social and economic cost to families and society [23]. SCI is a complex biological process that includes both primary and secondary damage and involves the nervous, immune, and vascular systems [24]. The initial mechanical trauma can lead to neuron necrosis and apoptosis, and the secondary damage often worsens the injury [25, 26]. Active research of SCI has made slow but consistent progress with respect to developing new treatments. With respect to mRNA and lncRNA, a recent study by Jin et al. [27] identified significant DEGs at 3 days, 2 weeks, and 1 month following SCI. Based on the results of Jin's study, we choose 3 days post-SCI as the time point of our study.

Our results demonstrated that the expressions of certain mRNAs and lncRNAs were dramatically changed 3 days after SCI. Furthermore, we identified 10 key genes in the injury group (group 2) and the rhEPO treatment group (group 3) that may play an important role in early acute phase of SCI. These genes may assist in further research of SCI and the development of new treatments.

The genes in the injury group (group 2) with significant changes in expression profiles were associated with the positive regulation of the immune response, regulation of vesicle-mediated transport, regulation of leukocyte activation, wound healing, regulation of transmembrane transport, and other significant biological processes. Previous studies have indicated that the primary cellular responses to SCI are inflammation and an immune response, which is consistent with our GO analysis results. SCI induces the activation of immune cells and inflammatory mediators, but the benefit of targeting the immune response to treat SCI is not clear [28].

Stimulation of the proliferation of leukocytes is also a key process of SCI that occurs from the immediate phase to the chronic repair phase. Our KEGG enrichment analysis demonstrated that the genes with changes of expression were involved in Epstein-Barr virus infection, focal adhesions, the calcium signaling pathway, retrograde endocannabinoid signaling, osteoclast differentiation, platelet activation, and SLE. In a prior study, KEGG enrichment analysis revealed that the toll-like receptor signaling pathway, p53 signaling pathway, MAPK signaling pathway, and Jak–STAT signaling pathway were related to SCI [29]. Obviously, our findings are not completely consistent with that of the prior study. We postulate that the different results may be because specimens were collected at different time points. Our PPI network analysis, however, identified FN1, PTPRC, CD44, CDC20, TYROBP, AURKB, TlR2, angiotensinogen, AGT, RAC2, and MMP9 as the top 10 high-degree hub nodes, suggesting these genes may play an indispensable role in the pathophysiological processes of SCI.

Our previous studies showed that EPO reduces apoptosis and inflammation and promotes myelin repair and functional recovery following compressive SCI in rats from the perspective of bioinformatics. Our prior results were the basis for performing the current study to identify genes differentially expressed after SCI, and after treatment with rhEPO. In the rhEPO treatment group (group 3), the DEGs were significantly associated with leukocyte chemotaxis, myeloid leukocyte migration, granulocyte migration, granulocyte chemotaxis, and neutrophil migration. These findings confirm that the inflammatory response and inflammatory cell activation play an indispensable role in the repair of SCI. A prior study showed that blocking inflammation via the administration of anti-inflammatory drugs can reduce inflammation and partially restore locomotor activity following SCI [30].

Our KEGG pathway analysis indicated that the most significant pathways associated with SCI and repair were cytokine-cytokine receptor interaction, chemokine signaling, and IL-17 signaling pathways. Previous studies have reported that cytokines play an important role in central nervous system (CNS) immune system interactions, and SCI can initiate immune responses characterized by the synthesis and release of chemokines and cytokines [31, 32]. In addition, an increase of IL-17 concentration can result in the increase in the size of a lesion after SCI. Study has shown that reducing the expression of IL-17 and IL-17-related inflammatory factors can protect neurons and promote recovery after SCI [33]. In the PPI network developed in this study, the top 10 high-degree hub nodes (Ccl4, Ppbp, Cxcl13, Ahsp, Ccl5, Alas2, Npy, Gng13, Ccl2, and Hba2.) were all chemokines, which are a superfamily of secreted proteins involved in immune-regulatory and inflammatory processes. Study has shown that CXCL13/CXCR5 signaling can promote diabetes-induced tactile allodynia through the production of proinflammatory cytokines in the spinal cord of male mice [34]. Additionally, Ppbp is a platelet-derived growth factor that belongs to the CXC chemokine family. Chio et al. [35] demonstrated that a traumatic brain injury can upregulate the expression of Ppbp in peripheral blood. Alas2 encodes a protein called heme that catalyzes the first step in the heme biosynthetic pathway and appears to promote a concurrent increase of neutrophilic meta-myelocytes and mature CD71 erythroid cells [36]. Furthermore, endogenous neuropeptide Y (NPY) and the activation of its associated receptors can exert long-lasting spinal inhibitory control of neuropathic pain [37]. We speculate that EPO may influence the expression of NPY to achieve behavioral NPY-induced antinociception. Taken together, the aforementioned studies and our results lead us to hypothesize that EPO plays an important role in the acute phase of SCI by regulating the inflammatory response and affecting the synthesis and release of inflammatory factors and/or chemokines.

To our knowledge, this is the first study that has used bioinformatics methods to investigate EPO and the treatment of SCI. While we identified DEGs and lncRNAs associated with SCI, and EPO treatment, there are some shortcomings of this study. First, the small numbers of specimens may affect the reliability of the results. However, we reduced individual differences by mixing different samples from the same group. While we identified DEGs, we did not explore their functions, nor did we explore the specific mechanisms of the lncRNAs identified. In the acute phase of SCI, primary injury can lead to neuron death, demyelination in the spinal cord, and eventually, axonal dieback. In this study, we only examined tissue specimens at 1 time point. Future studies should examine and compare specimens at multiple time points after SCI.

## 5. Conclusion

In conclusion, we identified differential expression profiles of mRNAs and lncRNAs in spinal cord samples in the subacute phase following SCI. We also identified DEGs between normal spinal cord and injured spinal cord and between injured spinal cord and SCI treated with rhEPO. Critical pathways affected by rhEPO treatment of SCI were also identified. These results may offer new insights into the cellular and pathophysiological processes involved in SCI and insights for the development of new treatment methods.

## Figures and Tables

**Figure 1:** In the volcano diagram, each point represents a gene, and the *X*-axis represents the logarithm of the multiple of the difference in expression of a certain gene in the two samples; the *Y*-axis represents the statistically significant negative logarithm of the gene expression change. The larger the absolute value of the *X*-axis, the greater the fold change in expression between the two samples; the larger value of *Y*-axis, the more significant the differential expression, and the more reliable the DEGs obtained by screening. The blue dots (fold change < −1) in the figure represent downregulated DEGs, the red dots (fold change > 1) represent upregulated DEGs, and the grey dots represent non-DEGs.

**Figure 2:** In the heatmap, the red color represents upregulated mRNAs or lncRNAs, and the blue color represents downregulated mRNAs or lncRNAs.

**Figure 3:** The qRT-PCR result was consistent with that of the microarray between group 3 and group 2, in that the first 3 mRNAs had a rising trend, while the last 3 mRNAs showed a downward trend. All 6 mRNA transcripts reached statistical significance (*p* < .05 for each mRNA, Student's *T* test), as seen in Figure 1. Verification expression levels of DEGs in qRT-PCR during EPO treatment of SCI in rats. DEGs: differentially expressed genes; SCI: spinal cord injury; EPO: erythropoietin.

**Figure 4:** GO term enrichment analysis of mRNAs in the early acute phase of SCI. (a) GO annotations of DEGs with top 15 enrichment scores between group 1 and group 2. (b) GO annotations of DEGs with top 15 enrichment scores between group 3 and group 1. The red represents BC; the green represents CC; the blue represents MF. BC: biological process; CC: cell component; MF: molecular function.

**Figure 5:** KEGG pathway analysis of DEGs in spinal cord samples in the subacute phase following SCI. (a) The top 15 KEGG analysis enrichment between group 2 and group 1. (b) The top 15 KEGG analysis enrichment between group 3 and group 2. The *X*-axis shows gene ratio, and the *Y*-axis shows the KEGG annotations. The larger the circle area, the more DEGs the pathway contains. KEGG: Kyoto Encyclopedia of Genes and Genomes.

**Figure 6:** Interaction of protein-protein network analysis of DEGs between group 2 and group 1. Nodes represent DEGs. Lines indicate interactions between DEGs.

**Figure 7:** Interaction of protein-protein network analysis of DEGs between group 3 and group 2. Nodes represent DEGs. Lines indicate interactions between DEGs.

**Table 1:** The list of primers for qRT-PCR.

Primer	Sequence (5′to 3′)
Actin b-F	GTGATGGACTCCGGAGACG
Actin b-R	GTGGTGAAGCTGTAGCCACG
Ccl5-F	GAAGATCTCCACAGCTGCATC
Ccl5-R	GTGACAAAGACGACTGCAAGG
Ppbp-F	CTTCAGACTCAGACCTACATC
Ppbp-R	CCACATTGTCACAGTGCGC
Ahsp-F	CTCATGCCTGAAGAAGACATG
Ahsp-R	CAGAATGATCCTGTATTTGGC
Plk5-F	GCACCACCGCAACATCGTG
Plk5-R	GGTCACCTATCTTAACTTCCATG
Mmp7-F	GGACTGCAGACATCATAATTGG
Mmp7-R	GTGGCCAAGTTCATGAGTGG
Esrp2-F	GGGATGACAAACCACTAGCTG
Esrp2-R	CTTGCCCTCTGGTATTCACTG

**Table 2:** The differential expression profile of the known mRNAs and lncRNAs.

Group	mRNA		lncRNA	
	Upregulation	Downregulation	Upregulation	Downregulation
G2 vs. G1	2471	1975	45	54
G3 vs. G2	151	76	9	5

The number of this table represented the quantity of differential expression of lncRNAs and mRNAs.

**Table 3:** The top 5 upregulated and downregulated lncRNAs between the group 2 and group 1.

Upregulated lncRNAs			Downregulated lncRNAs		
ID	log2FC	*p* value	ID	log2FC	*p* value
AABR07030791.1	8.19	8.50*E*-11	AABR07028797.1	-6.05	0.000167407
AABR07049503.1	6.02	0.000129838	AC105485.2	-5.86	0.000437654
AABR07027569.3	6.01	0.000152459	AABR07028793.1	-5.61	0.00116144
AABR07038983.1	5.84	2.00*E*-09	AABR07048040.1	-5.55	0.004700986
AABR07021998.1	5.77	0.000287606	AABR07007879.1	-5.33	0.005198832

**Table 4:** The top 5 downregulated and upregulated lncRNAs between the group 3 and group 2.

Upregulated lncRNAs			Downregulated lncRNAs		
ID	log2FC	p value	ID	log2FC	*p* value
LOC100910750	5.34	0.023054	AABR07069008.3	-5.09	0.019272
AC096330.1	4.02	0.033215	AABR07044454.1	-5.04	0.008021
AABR07002674.1	3.86	0.007318	AABR07062344.2	-4.32	0.031877
AABR07007055.1	2.42	0.015358	AABR07051515.2	-4.12	0.021149
AABR07019254.2	2.40	0.027412	AABR07053771.1	-2.42	0.025481

**Table 5:** The top 10 hub gene in the network between group 2 and group 1.

Rank	Name	Score	Rank	Name	Score
1	Fn1	108	6	Aurkb	61
2	Ptprc	85	7	Tlr2	60
3	Cd44	70	8	Agt	59
4	Cdc20	68	9	Rac2	58
5	Tyrobp	66	10	Mmp9	57

**Table 6:** The top 10 hub gene in the network between group 3 and group 2.

Rank	Name	Score	Rank	Name	Score
1	Ccl4	218	6	Alas2	121
2	Ppbp	193	7	Npy	120
3	Cxcl13	192	7	Gng13	120
4	Ahsp	127	9	Ccl2	106
5	Ccl5	125	10	Hba2	96

## Data Availability

No data were used to support this study.
